The article "Effect of HIV-1 Protease Inhibitor on IL-18 and IL-1β in Rats with Insulinoma" was retracted in 2023. Reasons: signs of a paper mill; suspected computer-generated content; unreliable results or conclusions; concerns about the data.

# Effect of HIV-1 Protease Inhibitor on IL-18 and IL-1*β* in Rats with Insulinoma

**DOI:** 10.1155/2022/1868749

**Published:** 2022-05-11

**Authors:** Haiying Lou, Luyong Guo

**Affiliations:** Department of Endocrinology, Zhuji People's Hospital of Zhejiang Province, Zhejiang 311800, China

## Abstract

This study is aimed at investigating the treatment effectiveness of HIV-1 protease inhibitor for rats with insulinoma and its effects on interleukin-1*β* (IL-1*β*) and interleukin-18 (IL-18). A total of 40 6-week-old nude mice were included in this study. We randomly assigned 20 rats for insulinoma modeling and divided them into model A and B groups. Another 20 rats were randomly divided into control A and B groups. Rats from the model A and control A groups were given HIV-1 protease inhibitors. The expression profiles of IL-18 and IL-1*β*, clinical indicators, water maze test results, oxidative stress damage, and changes in neurological functions in rats from each group were recorded. The expression levels of IL-18 and IL-1*β*, insulin level, the ratio of immunoreactive insulin to plasma glucose (IRI/G), escape latency, reactive oxygen species (ROS), and amyloid *β*-protein (A*β*) level were lower in the model A group than in the model B group while fasting blood glucose, platform crossing times, and superoxide dismutase (SOD) were higher in the model A group than in the model B group. The insulin level and hippocampus A*β* level were lower in the control A group than in the control B group. In contrast, other indicators in the control A group were not significantly different from those in the model B group. HIV-1 protease inhibitor is effective in the treatment of insulinoma in rats. It can significantly reduce IL-18 and IL-1*β* and protect the neurological functions in rats and has broad prospects for clinical application.

## 1. Introduction

An insulinoma is featured with excessive insulin secretion caused by an islet *β*-cell tumor or *β*-cell hyperplasia, posing a high risk of hypoglycemia [1]. Insulinomas are usually benign, with only 10.0-16.0% being malignant [2]. The present worldwide incidence of insulinoma is unclear, but it will attack people from any age group [3]. The most specific pathological change of insulinoma is the occurrence of hypoglycemia. In severe cases, patients may develop a certain degree of mental disorder, facing great significant threats to their everyday life [4]. The current incidence of insulinoma is not as high as malignant tumors such as gastric cancer and lung cancer. Still, its incidence increases yearly [5], with a significant potential threat. According to tumor progression, the existing principal clinical treatment of insulinoma is the surgical resection of pancreatic tissue [14], but invasive and traumatic surgery is detrimental, and the removal of pancreatic tissue adversely affects the patient's prognosis and life [6]. Conservative treatment regimens are available for a few patients unsuitable for the surgery, but they lead to a very long treatment cycle, with only a moderate cure rate [7].

Recent studies at home and abroad have proposed the essential role of targeted inhibitors in the future treatment of tumor diseases [8, 9]. Human immunodeficiency virus-1 (HIV-1) protease inhibitor is an antiretroviral drug to treat HIV infection, which can cause peripheral insulin resistance in HIV-infected patients [10]. We speculate that HIV-1 protease inhibitor may be effective for treating insulinoma. Although the incidence of insulinoma is not high, it can affect individuals from any age group and damage nerve functions, triggering clinical concerns [11]. Insulinoma should get treated as soon as possible in the early stages of disease progression, or it will cause irreversible damage to the brain [12]. Patients treated with radical surgery are prone to complications such as pancreatic fistulas, pseudopancreatic cysts, pancreatitis, and a high postoperative recurrence rate [13]. So, the search for an effective conservative treatment plan for insulinoma is of great significance. To verify our conjecture, we explored the therapeutic value of HIV-1 protease inhibitor for insulinoma, aiming to provide reference and guidance for the future treatment of insulinoma. Studies have shown that interleukin-1*β* (IL-1*β*) and interleukin-18 (IL-18) are closely related to the production of islet beta cells and nitric oxide (NO) [14, 15]; so, we measured the levels of IL-18 and NO to investigate the effect of HIV-1 protease inhibitor on insulinoma.

## 2. Materials and Methods

### 2.1. Basic Information on Rats

We purchased 40 clean 6-week-old nude mice from Beijing Vital River Laboratory Animal Technology Co., Ltd. (certificate number: SCXK (Beijing) 2016-0011). Rats were in a 1 : 1 sex ratio, weighing (210 ± 20) g. We raised rats in separate cages (5 rats per cage) at (29 ± 2) °C and 40-50% humidity and allowed their normal eating and light exposure. This study was carried out after getting approval from the Animal Ethics Committee of our hospital (approval number: ZJ No. 2019003548 (337)).

### 2.2. Methods

#### 2.2.1. Methods of Modeling

Animal modeling here was referred to in the study made by Collantes et al. [16]. We randomly assigned 20 of the 40 rats for diabetes modeling by giving them a one-time intraperitoneal injection of streptozotocin at a 180 mg/kg high dose. Then, tail blood was taken every three days to detect blood glucose. After six days, the modeling was considered successful if the blood glucose was over 20 mmol/L. Rat insulinoma INS-1 cell line purchased from BeNa Culture Collection (BNCC337862) was cultured to the logarithmic growth phase and digested by 0.025% trypsin before centrifuging. Then, the cell suspension was aspirated into the disposable scalp needle by a sterilized syringe and centrifuged by a hand centrifuge, with cells pushed to the pinhead. Successful rat models with diabetes were intraperitoneally injected with 3% sodium pentobarbital (2 mg/kg) for anesthesia. After anesthesia, the rats were placed prone for routine disinfection. An incision of approximately 1 cm was cut parallel from the left kidney to drag out the kidneys. Cells stored in the pinhead of the scalp needle were transplanted under the renal capsule, then the kidney was put back into the rat body, and the incision was sutured layer by layer.

#### 2.2.2. Experimental Methods

At 21 days after the modeling, nelfinavir (6.64 mg), the HIV-1 protease inhibitor, was dissolved in 200 *μ*L of 100% ethanol to prepare a solution at 50 mmol/L and placed in a refrigerator at -20°C for later use [17]. Successful rat models were randomly divided into model A and model B groups, while the other not modeled rats were randomly divided into control A and control B groups. Rats from model A and control A groups were injected with 4 ml of the HIV-1 protease inhibitor every seven days for four injections. We randomly selected five rats from each group before and after the infusion and sacrificed them by cervical dislocation under anesthesia to obtain the kidney tissues. Then, we photographed the melanoma metastases and counted them. Models with failed tumor transplantation were not included in the study results.

#### 2.2.3. Detection Method

Serum concentrations of IL-18 and IL-1*β* in rats from each group were measured by the enzyme-linked immunosorbent assay (ELISA). The IL-18 kit was provided by Beijing Lvyuan Bode Biotechnology Co., Ltd. (SEK50073) and the IL-1*β* kit by Suzhou Renold Biotechnology Co., Ltd. (ml001553). Clinical indicators were as follows: blood samples of rats were collected and sent to the laboratory of our hospital to detect the fasting blood glucose levels, insulin levels, and IRI/G before and after the treatment. Rats fasted for 12 hours before the blood draw. Water maze test was as follows: the water maze test was conducted 24 hours after the last injection of the HIV-1 protease inhibitor into rats.

The maze was 160 cm × 50 cm × 10 cm divided into four equal quadrants by two central perpendicular axes connected by four equidistant points marking *N*, *E*, *S*, and *W* on the wall. The platform was placed in any quadrant at 1 cm below the water containing the bleach at 25.0 ± 1.0°C. During the test, the external reference remained unchanged. Rats were placed in the maze facing the maze wall. Then, we recorded each rat's time finding the platform and climbing on it (escape latency). The training for finding the platform lasted for continuous five days, two sets of training daily (4 times of activity for one set, the interval was 5 minutes between two pieces of training and 4 hours between two sets). The water platform was removed on the 6th day, and rats were placed in the maze at the exact location facing the maze wall. The escape latency and the frequency of crossing the platform within 2 minutes of rats were recorded. Oxidative stress was as follows: on the 40th day of this experiment, we anesthetized all rats with an intraperitoneal injection of 3% sodium pentobarbital (2 mg/kg) and then sacrificed them to obtain the hippocampal tissues. Rats were dead when they stopped breathing, and the muscles were relaxed entirely, showing no responses to the tweezer clamping its tail.

The hippocampus tissues were collected and made into a tissue homogenate. The supernatant was obtained to detect SOD and ROS levels in the hippocampus. The SOD kit was purchased from Nanjing Jiancheng Bioengineering Institute (A001-1). The ROS kit was from Elabscience Biotechnology Co., Ltd. (E-BC-K138-F). Neurological function was as follows: according to the kit instructions, ELISA was used to detect A*β* levels in the hippocampus and rat serum. The A*β* kit was purchased from Linyi Aizelasi Biotechnology Co., Ltd. (EK-3332).

*(1) Assessment of Humane Endpoints*. Weight loss was as follows: a decrease in weight by 15-20% within two days, continuous absence of weight gain in the animals in the growth stage, or signs of cachexia or straight muscle wasting when the bodyweight is not monitored. Weakness was as follows: inability to access food and water, incapability to remain standing, or extreme difficulty standing for up to 24 hours. Please note that the liability of animals may also be due to the recovery from anesthesia. Organ infections were as follows: physical indicators and abnormal blood test results, poor treatment responses, and even progression to systemic diseases. Respiratory system dysfunction was as follows: severe respiratory infections, dyspnea, and cyanosis. Circulatory system dysfunction was as follows: severe anemia, uncontrolled bleeding (PVC less than 15%), and jaundice. Nervous system dysfunction was as follows: abnormal central nervous responses (twitching, trembling, paralysis, crooked head, etc.) and ineffective pain control. Others were as follows: persistent self-mutilation, nonhealing wounds, conditions that severely affect animals' ability to access food and water, end-stage infectious diseases, persistent hypothermia, significant organ, facial dysfunction, and behaviors and physiological phenomena occurring when animals suffer distress and pain.

### 2.3. Statistical Analysis

Statistical analysis was performed using SPSS24.0 statistical software (Shanghai Yuchuang Network Technology Co., Ltd.). Data visualization was performed using GraphPad 8 software (SOFTHEAD Inc.). The count data were expressed by the percentage (%) and compared in two groups by the chi-square test. The measurement data were represented by the mean ± standard deviation and compared between two groups by the *t*-test. The comparison between data before treatment and data after treatment was analyzed by the paired *t*-test. The comparison between multiple groups was performed using the one-way ANOVA and LSD post hoc test. The one-tailed *P* value less than *P* < 0.050 indicates statistical difference.

## 3. Results

### 3.1. Modeling Result

The modeling was successful in 19 (95.0%) of the 20 rats, with one death case during the modeling. We found obvious signs of bite on the dead rat, which suggests that the rat was attacked to death by other rats in the same cage. The final grouping situation was 10 in the model A group, 9 in the model B group, 10 in the control A group, and 10 in the control B group. The kidneys of nude mice transplanted with INS-1 cells showed clear signs of tumor formation, with uneven surface and a markedly larger size than normal kidneys. We noted obvious transplanted tumors in the collected left kidneys, which tested positive for insulin according to the immunohistochemical staining results.

### 3.2. Water Maze Test

The escape latency and platform crossing times between the control A and control B groups showed no difference (*P* = 0.782). Control A and control B groups had shorter escape latency and more platform crossing times than model A and B groups. The model B group had the most prolonged escape latency and the least number of platform crossings times among the four groups. More details are shown in Figure 1.

### 3.3. Comparison of IL-18 and IL-1*β* Levels

Before and after the treatment, the IL-18 and IL-1*β* level comparison showed no difference between control A and control B groups (*P* = 0.924). The comparison of IL-18 and IL-1*β* levels before treatment showed no difference between the model A group and model B group. At the same time, the IL-18 and IL-1*β* levels in the model A group were lower than those in model B and higher than those in control A and controlled B groups. After treatment, the IL-18 and IL-1*β* levels in control A and control B groups were not different from those before treatment. After treatment, the IL-18 and IL-1*β* levels decreased in the model A group but increased in the model B group (*P* < 0.050). More details are shown in Figure 2.

### 3.4. Comparison of Clinical Indicators

Before treatment, the comparison of fasting blood glucose, insulin, and IRI/G showed no difference between the control A and control B groups or between the model A and B groups. Before treatment, the model A and model B groups had lower fasting blood glucose and higher insulin and IRI/G than the control A and control B groups. The control A group was not different from the control B group in the fasting blood glucose and IRI/G before treatment but had lower insulin levels than the control B group. After treatment, the model A group had higher fasting blood glucose and lowered insulin and IRI/G than the model B group. The fasting blood glucose, insulin, and IRI/G in the control B group after treatment were not different from those before treatment. The insulin level in the control A group decreased after treatment (*P* < 0.050). The model A group had higher fasting blood glucose and lower insulin level and IRI/G after the treatment. The model B group had lower fasting blood glucose and higher insulin level and IRI/G after the treatment. More details are shown in Figure 3.

### 3.5. Comparison of Oxidative Stress

The comparison of SOD and ROS between the control A and control B groups showed no difference. Control A and control B groups had higher SOD and lower ROS than model A and model B groups. The model B group had the lowest SOD and the most elevated ROS among the four groups (*P* < 0.050). More details are shown in Figure 4.

### 3.6. Comparison of Neurological Function

The control A group was not different from the control B group in the serum A*β* level but had lower A*β* in the hippocampus than the control B group. The model B group had the highest serum and hippocampus A*β* among the four groups. More details are shown in Figure 5.

## 4. Discussion

Here, we analyzed the efficacy of HIV-1 protease inhibitor in rats with insulinoma, aiming to assess the clinical application value of HIV-1 protease inhibitor. In this study, rats from the model A group treated with HIV-1 protease inhibitor had lower IL-18 and IL-1*β* levels than rats from the model B group. IL-18 belongs to the IL-1 receptor family. It is abnormally expressed in insulitis and diabetes, playing an essential role in cytokine-mediated *β* cell destruction [18]. IL-18 is located in the 9th pair of chromosomes in mice, identified as one of the susceptible genes [19]. Insulinoma is also called islet *β*-cell tumor, and more than 50% of insulinoma are superficial *β*-cell tumors [20].

Therefore, in our study, IL-18 levels in rats from the model groups were much higher than those in the control groups. The reduction of the IL-18 level in the model A group after treatment indicates significant damage in the pancreatic *β* cells in insulinoma rats treated with HIV-1 protease inhibitor, which is one of the principles in selecting a drug for insulinoma treatment. IL-12 and IL-18 limit HIV-1 replication in primary macrophages by upregulating SAMHD1 [21], supporting that HIV-1 is related to IL-18 levels. The study by Falasca et al. [22] found that hypertriglyceridemia was closely related to serum ghrelin, adiponectin, and IL-18 levels in HIV-infected patients, further confirming the effect of HIV-1 protease inhibitor on IL-18. We hypothesize that one of the therapeutic mechanisms of HIV-1 protease inhibitor for insulinoma may be its inhibition on IL-18 level to reduce the destruction capacity of *β* cells. IL-1*β* is also a member of the IL-1 family, closely associated with pancreatitis, pancreatic cancer, and other diseases [23, 24]. When the pancreas gets damaged, the pancreatic cells can produce a large amount of IL-1*β*, induce the production of adhesion molecules, activate the accumulation of neutrophils in the cell tissue, and release oxygen free radicals, elastase, and proteolytic enzymes, causing tissue damage [25]. The markedly higher IL-1*β* levels can verify this in the model groups than in the control groups. The IL-1*β* level decreased in the model A group after the treatment, suggesting that the degree of pancreatic damage was reduced and the tissue became normal. Both HIV-1 and IL-1*β* can regulate the Fas ligand expression in human astrocytes via NF-*κ*B [26]. We hypothesize that the effect of HIV-1 protease inhibitor on IL-1*β* levels in the treatment of insulinoma may be achieved through the NF-*κ*B signaling pathway, but the present study did not conduct cell experiments to verify this, requiring in-depth analysis in our future research.

To further clarify the therapeutic effect of HIV-1 protease inhibitor on insulinoma, we measured the levels of relevant diagnostic indicators for insulinoma in each group of rats. Hypoglycemia is the most common concomitant disease of insulinoma. The detection of fasting blood glucose is critical for the primary diagnosis of insulinoma. A fasting blood glucose level of less than 2.78 mmol/L is clinically diagnosed as insulinoma [27]. The story of fasting blood glucose in rats from model groups met this diagnosis criterion before the treatment. It then increased after the treatment, proving the influential role of the HIV-1 protease inhibitor. The rise in the insulin level is a sign of impaired pancreatic function and a direct basis for diagnosing insulinoma [28]. IRI/G is more accurate than insulin in diagnosing insulinoma [29]. In this study, the IRI/G was higher in the model groups than in the control groups before the treatment, and the IRI/G has marked lower in the model A group than in the model B group after the treatment, suggesting that the IRI/G has observed lower in the model A group than in the model B group after the treatment, denoting that the HIV-1 protease inhibitor was effective in treating insulinoma. The insulin level decreased in the control A group after the injection with the HIV-1 protease inhibitor, indicating a promising prospect of HIV-1 protease inhibitor in lowering the insulin level.

Neurological impairment is one of the common complications of insulinoma. We conducted the water maze test and detected the levels of SOD, ROS, and A*β* in rat hippocampus to explore the effects of HIV-1 protease inhibitor on neurological function in rats. The results demonstrated that rats from the model A group had better performances in the water maze test, higher SOD, and lower ROS than those from the model B group. This may result from the effect of the HIV-1 protease inhibitor on IL-18 and IL levels. SOD and ROS are markers of oxidative stress. Oxidative stress injury results in overly produced ROS and excessive oxidation, causing tissue damage. The overly produced ROS not only directly attacks cell biofilms, induces apoptosis, or even causes necrosis but also works as a second messenger to activate nuclear transfer, thereby increasing the enzymatic activity of cysteinyl aspartate specific proteinase family members, causing damage to nerve cells, and promoting their apoptosis [30]. SOD can eliminate superoxide anion radicals produced during metabolism, which, being cytotoxic, can give rise to lipid peroxidation, damage to cell membranes, inflammation, tumorigenesis, and the development of autoimmune diseases [31]. The increase in SOD and the decrease in ROS in this study also indicate that the HIV-1 protease inhibitor causes more minor oxidative stress damages in rats, with extreme safety in its future clinical application. A*β* is an excellent reflection of nerve functions. It has been found to competitively bind the insulin to decrease the activity of insulin-degrading enzymes and induce insulin resistance [32]. The decrease in A*β* in the model A group after treatment also indicated improved insulin function and nerve function of rats, demonstrating the clinical value of the HIV-1 protease inhibitor. In this study, rats from the control A group injected with HIV-1 protease inhibitor showed no signs of deterioration in those relevant indicators but had decreased insulin and A*β* levels, suggesting that HIV-1 protease inhibitors do not harm the average human body, enjoying excellent application value.

The aim of this study was to investigate the therapeutic effect of HIV-1 protease inhibitors on insulinoma. Due to the limited experimental conditions, we have not determined the mechanism of action of HIV-1 protease inhibitor in the treatment of insulinoma; so, the mechanism of treatment of insulinoma needs to be studied in the future. Considering the difference between animal experiments and human experiments, we will conduct human experiments in the next study to confirm the applicability of HIV-1 protease inhibitors to humans. In the future, we will conduct in-depth and comprehensive analysis on the above deficiencies to obtain the most accurate results. In summary, HIV-1 protease inhibitor has marked treatment effectiveness for rats with insulinoma. It can significantly reduce IL-18 and IL-1*β* and protect the neurological functions in rats, enjoying a promising prospect in its clinical application.

## Figures and Tables

**Figure 1:** Results of water maze test. (a) Comparison of the escape latency. (b) Comparison of the frequency of platform crossing. “^∗^” indicates *P* < 0.050 when compared with the model A group; “#” indicates *P* < 0.050 when compared with the model B group.

**Figure 2:** Comparison of IL-18 and IL-1*β* levels. (a) Comparison of the IL-18 level before and after treatment. (b) Comparison of the IL-1*β* level before and after treatment. “^∗^” indicates *P* < 0.050 when compared with the model A group at the same time; “#” indicates *P* < 0.050 when compared with the model B group at the same time; “&” indicates *P* < 0.050 when compared with the levels before treatment in the same group.

**Figure 3:** Comparison of clinical indicators. (a) Comparison of the fasting blood glucose before and after treatment. (b) Comparison of the insulin level before and after treatment. (c) Comparison of the IRI/G before and after treatment. “^∗^” indicates *P* < 0.050 when compared with the model A group at the same time; “#” indicates *P* < 0.050 when compared with the model B group at the same time; “&” indicates *P* < 0.050 when compared with the levels before treatment in the same group.

**Figure 4:** Comparison of oxidative stress. (a) Comparison of the SOD. (b) Comparison of the ROS. “^∗^” indicates *P* < 0.050 when compared with the model A group; “#” indicates *P* < 0.050 when compared with the model B group.

**Figure 5:** Comparison of neurological functions. (a) Comparison of the A*β* level in serum. (b) Comparison of the A*β* level in the hippocampus. “^∗^” indicates *P* < 0.050 when compared with the model A group; “#” indicates *P* < 0.050 when compared with the model B group; “&” indicates *P* < 0.050 when compared with the control A group.

## Data Availability

The datasets used and/or analyzed during the current study are available from the corresponding author on reasonable request.
